The article "Identification of a Novel Risk Model: A Five-Gene Prognostic Signature for Pancreatic Cancer" was retracted in 2023. Reasons: unreliable results or conclusions; concerns about the data; concerns about the peer review; concerns about the citations.

# Identification of a Novel Risk Model: A Five-Gene Prognostic Signature for Pancreatic Cancer

**DOI:** 10.1155/2022/3660110

**Published:** 2022-07-08

**Authors:** Xiaoguang Wang, Man Ni, Daxiong Han

**Affiliations:** School of Pharmaceutical Sciences, Xiamen University, Xiamen 361102, China

## Abstract

**Objective:**

Biomarkers for pancreatic cancer (PCa) prognosis provide evidence for improving the survival outcome of this disease. This study aimed to identify a prognostic risk model based on gene expression profiling of microarray bioinformatics analysis.

**Methods:**

Prognostic immune genes in the TCGA-PAAD cohort were identified using the univariate Cox regression and Kaplan–Meier survival analysis. Multivariate Cox regression (stepAIC) was used to identify prognostic genes from the top 20 hub genes in the protein-protein interaction (PPI) network. A prognostic risk model was established and its performance in predicting the overall survival in PCa was validated in GSE62452. Gene mutations and infiltration immune cells in PCa tumors were analyzed using online databases.

**Results:**

Univariate Cox regression and Kaplan–Meier survival analyses identified 128 prognostic genes. Multivariate Cox regression (stepAIC) identified five prognostic genes (PLCG1, MET, TNFSF10, CXCL9, and TLR3) out of the 20 hub genes in the PPI network. A prognostic risk model was established using the signature of five genes. This model had moderate to high accuracies (AUC > 0.700) in predicting 3-year and 5-year overall survival in TCGA and GSE62452 cohorts. The Kaplan–Meier survival analysis showed that high-risk scores were correlated with poor survival outcomes in PCa (*p* < 0.05). Also, mutations in the five genes were related to poor survival. The five genes were related to multiple immune cells.

**Conclusions:**

The prognostic risk model was significantly correlated with the survival in PCa patients. This model modulated PCa tumor progression and prognosis by regulating immune cell infiltration.

## 1. Introduction

Pancreatic adenocarcinoma (PAAD/PCa) is estimated to be the second cause of cancer-related deaths worldwide in the next 10 years [1, 2]. The mortality of PCa-related death has increased from over 200,000 cases in 2005 to over 432,000 cases in 2018 [3, 4]. Also, the 5-year survival rate of PCa is as low as 10%, with a little change over the last few decades [2, 5, 6]. Therefore, there is an increasing demand for efficient and reliable biomarkers for the early diagnosis and prognosis evaluation of PCa. A number of preclinical and clinical studies showed that many diagnostic and prognostic biomarkers promote the early diagnosis of cancers, improve cancer treatment, or contribute to the development of personalized treatment [7, 8]. Although some biomarkers have not been approved clinically or certified extensively, many studies have shown the potential value in clinical application. Also, the advances in bioinformatics techniques and development in analytical tools promote the identification of marker genes. Microarray techniques allow the identification of mass biomarkers by exploring gene expression profiling and molecular mechanisms related to tumor progression or prognosis [9–12].

For instance, the chaperonin-containing TCP1 subunit 6A (CCT6A) gene was identified to be a prognostic biomarker in breast cancer [10]. Its expression was markedly related to poor survival. CCT6A was correlated with the cell cycle and the expression of CCNA2/B2. Moreover, several studies showed that CCT6A was associated with the prognosis of hepatocellular carcinoma [13], colorectal cancer [14], cervical cancer [15], glioblastoma [16], and Ewing sarcoma [17]. Sun et al. [14] showed that CCT6A was correlated with decreased immune infiltrates. Besides, there is increasing evidence showing that immune cell infiltration plays a vital role in the disease progression by regulating tumor microenvironment or immunosuppression [18, 19]. For instance, CXCL5 was related to poor survival in PCa and contributed to tumor-infiltrating immune suppressive cells in PCa cells, including M2 macrophages and neutrophils [20]. These results show that immunity plays a crucial role in tumor development and prognosis. Nevertheless, very few of immune-related genes of PCa have been investigated for the early diagnosis or prognosis, and the identification of novel biomarkers of PCa is urgently needed.

In this study, we employed bioinformatics and microarray analysis to identify prognostic immune-related genes in PCa. Besides, a prognostic risk model was established to illustrate the prognostic value of these genes. Our study may further uncover the molecular mechanism of PCa and provide a novel prognostic strategy for PCa.

## 2. Materials and Methods

### 2.1. Data Collection

The PCa gene expression microarray dataset (GSE62452) was downloaded from the Gene Expression Omnibus (GEO) database (https://www.ncbi.nlm.nih.gov/geo/). The dataset (GPL6244, (HuGene-1_0-st) Affymetrix Human Gene 1.0 ST Array) consisted of samples collected from 65 PCa patients (16 alive and 49 dead). The PCa gene expression RNA-seq in the *Cancer* Genome Atlas (TCGA; FPKM value; 84 alive and 92 dead) was downloaded from the UCSC Xena website (https://xenabrowser.net/datapages/).

### 2.2. Data Preprocessing

The hugene 10 sttran script cluster. Db package was used for data preprocessing of the GSE62452 dataset. The TCGA data processing was performed using the *R* package. Gene (protein_coding) annotation was conducted in the HUGO Gene Nomenclature Committee (HGNC; https://www.genenames.org/) database.

### 2.3. Identification of Prognostic Genes

Univariate Cox regression analysis was performed to identify prognostic genes. The significant criterion was set as *p* value <0.01. Also, the immune-related genes were identified in the Immunology Database and Analysis Portal (ImmPort; https://www.immport.org/home). Common genes between TCGA annotated genes and the ImmPort database were identified. Then, the *R* survival [21] and survminer [22] packages were used to perform survival analysis (the Kaplan–Meier method) for common genes. Immune genes with the independent prognostic ability (log rank *p* < 0.05) were regarded as prognostic genes.

### 2.4. Construction of the Protein-Protein Interaction (PPI) Network

The PPI interaction pairs across prognostic genes were identified and downloaded from the STRING database (version 11.5; https://cn.string-db.org/cgi/input.pl). Construction of the PPI network was performed using the Cytoscape (version 3.8.0; https://apps.cytoscape.org). Also, the cytoHubba plugin was used to identify the hub nodes (top 20) in the PPI network.

### 2.5. Construction and Assessment of the Prognostic Risk Model

The stepAIC algorithm [23] was a stepwise logistic regression method. We used the stepAIC algorithm to identify prognostic genes in the top 20 hub nodes (multivariate Cox regression analysis) and construct a prognostic risk model. The receiver operating characteristic (ROC) curve was constructed using the pROC package [24] for each gene to evaluate their prognostic value. The prognostic risk score (PRS) of each sample was calculated using the model. Then, the samples in both datasets (TCGA and GSE62452) were divided into high-risk and low-risk groups based on risk scores (cutoff). The Kaplan–Meier method in the survminer [22] and survival [21] packages in *R* were used for survival analysis.

The correlations of PIS with clinical variables in the TCGA dataset were analyzed using the multivariate Cox regression analysis. The ggforest method in *R* survminer was used to construct the forest plot.

### 2.6. Identification of Differentially Expressed Genes (DEGs) between High-Risk and Low-Risk Groups

The DEGs between high-risk and low-risk groups in the TCGA dataset were identified using the Limma package (version 3.34.0; https://bioconductor.org/packages/release/bioc/html/limma.html). DEGs were screened out using the criteria of adjusted *p* value <0.05 and |log_2_ (Fold change, FC) ≥ 0.5. The pheatmap (version 1.0.8; https://cran.r-project.org/package=pheatmap) in *R* was used to perform hierarchical clustering of DEGs.

### 2.7. Functional Enrichment Analysis

Gene Ontology (GO) biological process, cellular component, molecular functions, and Kyoto Encyclopedia of Genes and Genomes (KEGG) pathways related to prognostic genes or DEGs were identified using the Metascape tool (https://metascape.org/gp/index.html), with the following criteria: *p* < 0.05, minimum count = 3, and enrichment factor >1.5. Also, the gene set enrichment analysis (GSEA) methods were performed for genes. The reference genomes were “c2.cp.kegg.v7.4.symbols.gmt,” “c5.go.bp.v7.4.symbols.gmt,” “c5.go.mf.v7.4.symbols.gmt,” and “c5.go.cc.v7.4.symbols.gmt.” The criterion for the significant items of GSEA was set as *p* < 0.05. The clusterProfiler package [25] was used to show the results.

### 2.8. Analysis of Mutations in Genes in the Prognostic Risk Model

The cBioPortal (https://www.cbioportal.org) is a publicly available database used for the interactive exploration of multiple cancer genomics datasets. The mutations in genes in the prognostic risk model were identified in cBioPortal. Then, the correlations of mutations with the clinicopathologic characteristics and survival data in the TCGA-PAAD cohort were analyzed using the Kaplan–Meier survival analysis.

### 2.9. Infiltrating Immune Cells in PCa

The cell type identification by estimating relative subsets of RNA transcripts (CIBERSORT) [26] enables the estimation of the abundances of 22 immune cell types using gene expression data. The correlations between gene expression patterns and the abundances of immune cells were analyzed using the corrplot package in *R* [27].

## 3. Results

### 3.1. Screening of Prognostic Immune-Related Genes

A total of 17,273 genes were identified in the TCGA-PAAD data in the HGNC database. Then, 3,427 genes were found to be notably associated with the survival status in PCa patients by univariate Cox regression analysis, including 216 immune-related genes. To select genes having independent prognostic significance for PCa from the 216 immune-related genes, the Kaplan–Meier survival analysis was applied. The Kaplan–Meier survival analysis showed that 128 genes were independent risk factors for the overall survival of PCa (Table S1). To explore the underlying molecular functions of the 128 genes mentioned above, GO and KEGG pathway enrichment were analyzed. Functional enrichment analysis showed that these genes were associated with GO categories including “GO : 0048018: receptor-ligand activity,” “GO : 0070851: growth factor receptor activity,” and “GO : 005179: hormone activity.” Also, these genes were related to KEGG pathways, including “hsa04060: cytokine-cytokine receptor interaction,” “hsa04510: Focal adhesion,” and “hsa04210: Apoptosis” (Figure 1(a)).

### 3.2. Selection of Hub Genes Based on the PPI Network

To ascertain the interplay among the 128 genes, the PPI network was established by means of the STRING database and cytoscape software. According to Figure S1, the PPI network of these genes consisted of 113 nodes (gene products) and 385 edges (interaction pairs). To further screen the significant genes from these 128 genes, the cytoHubba plugin was applied for screening of hub genes. As shown in Figure 1(b), a total of 20 candidate hub genes were screened out and some of them were related to chemokines and their receptors, such as CXCL9, CXCL10, and CXCL11.

### 3.3. Determination of Independent Prognostic Indicators Based on a Prognostic Risk Model

To screen vital prognostic genes from the 20 hub genes presented above, the multivariate Cox regression analysis model was employed. Consequently, five genes were identified as independent prognostic markers, including phospholipase C*γ*1 (PLCG1; HR = 0.31, *p* < 0.001) MET proto-oncogene, receptor tyrosine kinase (MET; HR = 1.90, *p* < 0.001), TNF superfamily member 10 (TNFSF10; HR = 1.36, *p*=0.051), C-X-C motif chemokine ligand 9 (CXCL9; HR = 1.28, *p* < 0.001), and toll-like receptor 3 (TLR3; HR = 0.66, *p*=0.066) (Figure 2). Then, to further validate the prognostic importance of the 5 identified prognostic genes, a prognostic risk model was established for risk and survival evaluation. The ROC curve demonstrated that these five genes had moderate AUC values (AUC > 0.500) in predicting the survival status of PCa (Figure 3(a)). Also, the results showed that the patients with high expression levels of CXCL9, MET, TNFSF10, and TLR3 in PCa tumor tissues had lower survival probabilities than those who had low expression levels of these genes (log rank *p* < 0.05; Figures 3(b)–3(e)). Meanwhile, the patients with low PLCG1 expression levels in PCa tumor tissues showed poorer survival in comparison to those with high PLCG1 expression levels (log rank *p*=0.0053; Figure 3(f)).

### 3.4. Validation of the Prognostic Risk Model

To further verify the prognostic risk model for PCa, the PCa patients in the TCGA and GSE62452 datasets were divided into the high-risk and low-risk groups according to the PRS, and survival probabilities in each group were assessed. The Kaplan–Meier survival analysis demonstrated that the patients in the high-risk group showed notable lower survival probabilities than those in the low-risk group (log rank *p* < 0.05; Figures 4(a)-4(b)). Also, time-dependent ROC curve analysis was performed to assess the prognostic risk model. According to the results, the prognostic risk model has moderate to high accuracies (AUC > 0.700) in predicting 3-year and 5-year survival status in both TCGA and GSE62452 datasets (Figures 4(c)-4(d)).

To explore the potential prognostic clinical factors of PCa, the multivariate Cox regression analysis model was applied.  Figure 5(a) shows that the PRS of TCGA-PAAD patients was significantly associated with the patients' ages(HR = 1.02, *p*=0.071). To determine whether age affects the survival of PCa patients, the patients were assigned into “Age ≤ 65” and Age > 65 groups, and the survival probabilities were evaluated in each group. The results demonstrated that the survival probabilities of the patients were negatively related to the PRS in both age groups (*p* < 0.05).

To investigate the underlying molecular mechanism of the DEGs in PCa, the prognostic risk model was used, and GO term and KEGG pathway analysis was performed. We identified 654 DEGs between tumors in the high-risk and low-risk groups in TCGA-PAAD patients. As shown in Table 1, these genes were associated with pathways including “focal adhesion,” “axon guidance,” “cell cycle,” “ECM receptor interaction,” and “P53 signaling pathway.” The result of clusterProfiler functional enrichment analysis is shown in Table S2. Most of the DEGs were related to cell-cell interaction, adhesion, and junction.

### 3.5. Mutations in Five Prognostic Genes

To determine the connection between mutations in the prognostic genes and overall survival in PCa, the mutations of these genes were identified and overall survival probabilities of the patients were assessed. The cBioPortal online database showed that the MET gene had the highest mutation rate (9%) among samples, followed by TNFSF10 (7%), PLCG1 (5%), CXCL9 (5%), and TLR3 (3%). Furthermore, the results showed that the patients in gene-mutated status had low probabilities of overall survival (log rank *p*=5.81*e* − 05; Figure 6(a)) and disease-free survival (log rank *p*=5.88*e* − 03; Figure 6(b)).

### 3.6. Immune Cell Infiltration in the TCGA-PAAD Cohort

To explore PCa tumor immune correlation of the five prognostic genes, the immune/infiltrating cells in the tumor tissues were assessed. The CIBERSORT algorithm showed that the five prognostic genes were positively correlated with multiple immune cells (Figure 7(a)). For instance, the CXCL9 and MET genes were positively associated with M1 macrophages and activated/memory CD4 T cells, and CXCL9 and TLR3 genes were positively associated with gamma delta (*γδ*) T-cells. Also, we found that PCa tissues with high PRSs had higher percentages of M1/M0 macrophages and neutrophils compared with those who had low PRSs (Figure 7(b)).

## 4. Discussion

PCa is a deadly and aggressive disease with a rising mortality rate in both genders owing to deficiencies in early diagnosis and efficient treatment [28, 29]. At present, radical surgical resection is regarded as the standard and most effective remedy. However, the recurrence rate of PCa is pretty high [30, 31]. Molecular biomarkers are a typically strategy for prognosis evaluation of diseases. Furthermore, evidence has demonstrated that molecular biomarkers, such as CA19-9 [32] and Cripto-1 [33], can be targets of PCa prognosis. Regretfully, these biomarkers have insufficient sensitivity, and PCa remains largely incurable. Hence, more effective biomarkers for the prognosis evaluation of PCa are desperately required.

The immune system plays a vital role in the development and progression of human cancer. [34, 35] Accumulating evidence shows that immunotherapy has become a potent clinical strategy for treating malignancies, such as multiple myeloma (MM) [36] and melanoma [37]. Previous research indicates that immunotherapy may be a promising strategy for PCa [38]. Recently, immune-related genes, such as FN1 and ANXA1, have been identified as prognostic indicators of PCa [39]. Nevertheless, the prognostic significance of these genes needs to be further verified. In our study, 216 immune-related genes were found to be associated with the development and progression of PCa by bioinformatic analysis. Among these genes, 128 immune-related genes showed a significant prognostic value for PCa via overall survival analysis. Then, 20 hub genes were screened out from the PPI network and most of them were linked with chemokines and their receptors, including CXCL9. Among the 20 hub genes, 5 immune-related genes (PLCG1, MET, TNFSF10, CXCL9, and TLR3) showed a moderate value in predicting the survival status of PCa.

A number of studies showed that the five genes described above were associated with the prognosis, progression, development, and treatment response of a wide variety of tumors, including small cell lung cancer [40], lower-grade gliomas [41], PCa [42, 43], prostate cancer [44], clear cell renal cell carcinoma [45, 46], and stomach adenocarcinoma [47]. For instance, TLR3 expression was positively correlated with survival time in stomach adenocarcinoma [47]. Li et al. [41] showed that the low PLCG1 level was correlated with a good survival status in patients with lower-grade gliomas. Besides, the inhibition of PLCG1 suppressed the growth of small cell lung cancer cells by acting as an effector of FGFR1 signaling [40]. Also, a high level of CXCL9 was significantly related to a better survival outcome in patients with advanced PCa [43]. Gao et al. [42] showed that CXCL9 supplementation promoted the progression of tumors in a mouse model. According to survival analysis, the expression levels of MET, TNFSF10, CXCL9, and TLR3 were negatively related to the survival probabilities of patients with PCa, while the expression level of PLCG1 is positively related to the survival probabilities. Then, the five-gene prognostic risk model was constructed. Consequently, we found that the survival probabilities of patients in the low-risk group were notably higher than those of patients in the low-risk group. Meanwhile, the prognostic risk model showed moderate to high accuracies in the prognostic prediction for PCa patients based on TCGA and GSE62452 cohorts. Taken together, these results imply that PLCG1, MET, TNFSF10, CXCL9, and TLR3 may be vital prognostic indicators of PCa.

Gene mutations are known to play a crucial part in tumor progression [48]. A body of evidence showed that gene mutations can be prognostic indicators of tumors and cancers [49–51]. For example, FREM2 [48], CSMD1 [52], and ARID1A [53] mutations, have been identified as potential prognostic biomarkers of colorectal cancer, gastric cancer, and hepatocellular carcinoma, respectively. Furthermore, there is evidence showing the association of genetic mutations in TLR3, TNFSF10, and MET, with the risk and survival of human cancer [54–56]. Gray et al. [57] showed that TLR3 polymorphisms (rs3775291) were associated with poor overall survival in patients with colorectal cancer. Also, the polymorphisms in TNFSF10 (rs1131568 and rs1131579) were related to low survival rates and high recurrence rates in patients with hepatocellular carcinoma [54]. According to the mutation analysis, PLCG1, MET, TNFSF10, CXCL9, and TLR3 showed a mutational status in PCa in different degrees. Also, the results demonstrated that the mutational status in the five genes was correlated to poor survival in PCa. These results suggest that the mutations of the five genes may be a prognostic signature of PCa.

There is plenty of evidence showing the associations of the PLCG1, TLR3, and CXCL9 genes with immune infiltration in tumor microenvironment [42, 45, 47, 58, 59]. These genes were associated with the prognosis of tumors by regulating the abundance of tumor-infiltrating dendritic cells, macrophages, neutrophils, natural killer (NK) cells, B cells, and T cells [42, 45, 47, 59, 60]. TLR3 has been identified to be associated with the infiltration of immune cells, including dendritic cells, macrophages, neutrophils, NK cells, B cells, and T cells, in the renal clear cell carcinoma [45]. Also, the TLR3 expression level in stomach adenocarcinoma was correlated with the abundance of immune cells [47]. A preclinical research study of a mouse PCa model showed that CXCL9 supplementation promoted tumor progression by reducing tumor-infiltrating CD8+ cytotoxic T lymphocytes [42]. CXCL9 is a marker of M1 macrophages [61]. Tumor-infiltrating M1 and M2 macrophages were both associated with survival in cancer patients [62, 63]. M1 macrophages are commonly considered proinflammatory and antitumor [64, 65]. Wang et al. [66] showed that decreased tumor-infiltrating M1 macrophages reduced the overall survival of patients with ovarian cancer. Our present study showed that the five genes were associated with the infiltration of multiple immune cells, including M1 macrophages, T cells, and dendritic cells. These results indicate that the five prognostic immune genes play crucial roles in the progression and prognosis of PCa by regulating the microenvironment in PCa tumor cells.

## 5. Conclusions

Our present study established a prognostic risk model of five prognostic immune genes (PLCG1, MET, TNFSF10, CXCL9, and TLR3). The five genes and prognostic risk model were significantly correlated with the survival status in PCa. The five genes were associated with the progression of PCa tumors by regulating the infiltration of immune cells. In our study, we have identified a five-gene prognostic signature for PCa and may provide novel therapeutic targets for PCa. Nevertheless, a large cohort trial study should be performed to further validate the potential value of the risk model in PCa prognosis.

## Figures and Tables

**Figure 1:** Functional enrichment analysis for prognostic genes (a) and 20 hub genes (b). (a): The top 20 terms (Gene Ontology terms and KEGG pathways) associated with the 128 immune-related genes based on overall survival of TCGA-PAAD patients. (b): The 20 hub genes and interactions in the protein-protein interaction network. Color depth corresponds to interaction degree/score by the cytoHubba plugin in cytoscape. Orange and red colors denote low and high scores, respectively.

**Figure 2:** The forest plot of the hazard ratios presenting the results of multivariate Cox regression analysis for identification of independent prognostic indicators.

**Figure 3:** Survival analysis of the genes in prognostic risk model. (a): The receiver operating characteristic (ROC) curves of five prognostic genes in the TCGA dataset. AUC, area under ROC. (b)–(f): Kaplan–Meier survival analysis for the five prognostic genes in the TCGA dataset.

**Figure 4:** Assessment of the prognostic risk model in pancreatic cancer. (a) and (b): The results of Kaplan–Meier survival analysis in the TCGA and GSE62452 dataset, respectively. (c) and (d): The time-dependent receiver operating characteristic (ROC) curves of the model in the TCGA and GSE62452 dataset, respectively. AUC, area under ROC. FP, false positive rate. TP, true positive rate. Clinical variables associated with PRS in PCa.

**Figure 5:** Clinical factors correlated with a prognostic risk score in the TCGA-PAAD cohort. (a): The forest plot indicating the results of multivariate Cox regression analysis of clinical factors related to prognostic risk scores. HR, hazard ratio. CI, confidence interval. (b) and (c): the Kaplan–Meier survival analysis in TCGA-PAAD patients with different age groups. DEGs between high-risk and low-risk PCa tumors.

**Figure 6:** Survival analysis for patients based on the gene mutational status. Gene mutational status was identified from the cBioPortal online database. (a) and (b): Kaplan–Meier survival curves of overall survival and disease-free survival in TCGA patients with different mutational statuses, respectively.

**Figure 7:** Immune cell infiltration analysis based on the five prognostic genes. (a) correlation of gene expression patterns with the abundances of 22 immune cell types. Blue and red color denote negative and positive correlation, respectively. (b) Cell composition of 22 immune cells in PCa tumors with high- and low-risk scores. ^*∗*^ and ^*∗∗*^, *p* < 0.05 and 0.01, respectively.

**Table 1:** KEGG pathways (top 20) associated with the differentially expressed genes between TCGA-PAAD tumor tissues with high and low prognostic risk scores.

Description	Set size	ES	NES	*p* value
KEGG_PATHWAYS_IN_CANCER	320	−0.45	−1.87	1.29E − 03
KEGG_REGULATION_OF_ACTIN_CYTOSKELETON	206	−0.44	−1.76	1.39E − 03
^*∗*^KEGG_FOCAL_ADHESION	199	−0.48	−1.90	1.40E − 03
^*∗*^KEGG_AXON_GUIDANCE	128	−0.44	−1.65	1.49E − 03
KEGG_TIGHT_JUNCTION	129	−0.49	−1.84	1.49E − 03
KEGG_SYSTEMIC_LUPUS_ERYTHEMATOSUS	110	−0.50	−1.85	1.51E − 03
KEGG_CELL_CYCLE	124	−0.55	−2.02	1.53E − 03
KEGG_PYRIMIDINE_METABOLISM	95	−0.42	−1.50	1.54E − 03
KEGG_SMALL_CELL_LUNG_CANCER	84	−0.55	−1.95	1.59E − 03
^*∗*^KEGG_ECM_RECEPTOR_INTERACTION	82	−0.61	−2.13	1.59E − 03
KEGG_ARRHYTHMOGENIC_RIGHT_VENTRICULAR_CARDIOMYOPATHY_ARVC	74	−0.51	−1.77	1.63E − 03
KEGG_ADHERENS_JUNCTION	73	−0.56	−1.94	1.64E − 03
KEGG_PANCREATIC_CANCER	70	−0.53	−1.81	1.64E − 03
KEGG_ANTIGEN_PROCESSING_AND_PRESENTATION	67	−0.56	−1.91	1.64E − 03
^*∗*^KEGG_P53_SIGNALING_PATHWAY	68	−0.53	−1.79	1.66E − 03
KEGG_PATHOGENIC_ESCHERICHIA_COLI_INFECTION	54	−0.59	−1.93	1.68E − 03
KEGG_GLYCOLYSIS_GLUCONEOGENESIS	57	−0.52	−1.69	1.70E − 03
KEGG_PROTEASOME	43	−0.71	−2.17	1.73E − 03
^*∗*^KEGG_O_GLYCAN_BIOSYNTHESIS	29	−0.60	−1.71	1.75E − 03
KEGG_BLADDER_CANCER	42	−0.62	−1.89	1.76E − 03

NES, normalized enrichment score. ES, enrichment score. ^*∗*^overlapping pathways between GSEA and clusterProfiler functional enrichment analysis.

## Data Availability

The data used to support the findings of this study are available from the corresponding author upon request.

## Supplementary Materials

Supplementary Materials Table S1: The 128 independent risk factors for overall survival of pancreatic cancer (prognostic genes). Figure S1: The protein-protein interaction (PPI) network of 128 prognostic genes in pancreatic cancer. Color depth and node size corresponds to interaction degree. Orange and blue colors note low and high degree, respectively. Table S2: Functional enrichment analysis result (top 10 terms) of the differentially expressed genes between TCGA-PAAD tumor tissues with high and low prognostic risk scores.
